# Land use land cover change as a casual factor for climate variability and trends in the Bilate River Basin, Ethiopia

**DOI:** 10.1371/journal.pone.0311961

**Published:** 2024-12-31

**Authors:** Samuel Shibeshi Bikeko, Dr. E. Venkatesham

**Affiliations:** Department of Geography, Central University of Tamil Nadu, School of Earth Sciences, Thiruvarur, Tamil Nadu, India; Mattu University, ETHIOPIA

## Abstract

Land use and land cover (LULC) changes are crucial in influencing regional climate patterns and environmental dynamics. However, the long-term impacts of these changes on climate variability in the Bilate River Basin remain poorly understood. This study examines the spatiotemporal changes in LULC and their influence on climate variability in the Bilate River Basin, Ethiopia, over the period from 1994 to 2024. Utilizing multispectral satellite imagery from Landsat 5, 7, and 8, along with meteorological data from five stations, LULC was classified using the Random Forest algorithm on the Google Earth Engine platform. Climate variability and trends were assessed using the Mann-Kendall trend test, the Standardized Precipitation Index (SPI), and the Standardized Temperature Index (STI). The results reveal a consistent decline in forest cover, with a rapid annual loss of 4,681.2 hectares between 2014 and 2024. Concurrently, agricultural land expanded at an annual rate of approximately 1,141 hectares, while urban areas grew by 24.3 hectares annually in recent years. These LULC changes have contributed to significant climate variability in the region. The upper catchment experienced notable declines in rainfall and warming across all seasons. In the middle catchment, spring rainfall increased, accompanied by moderate summer warming. The lower catchment saw significant increases in spring and autumn rainfall, with no notable temperature trends. These findings highlight the critical impact of LULC changes on the region’s climate and emphasize the need for sustainable land management and conservation practices to address deforestation, urbanization, and agricultural expansion.

## 1. Introduction

Land Use and Land Cover Change (LULCC) significantly contributes to climate change through various mechanisms, including deforestation [1], agricultural expansion [2], urbanization [3], and the degradation of wetlands and grasslands [4]. Deforestation releases stored carbon dioxide (CO2) into the atmosphere, with studies indicating that it accounts for about 10–15% of global anthropogenic CO2 emissions [5,6]. The conversion of natural landscapes into agricultural lands leads to substantial greenhouse gas (GHG) emissions, particularly methane (CH4) and nitrous oxide (N2O) from livestock and rice paddies [7,8]. Urbanization increases local temperatures through the heat island effect and boosts GHG emissions due to higher energy [9,10]. Draining wetlands and degrading peatlands result in the oxidation of stored organic matter, releasing CO2 and CH4 [11,12]. Additionally, the conversion of grasslands and shrublands disrupts carbon and water cycles, reducing biodiversity and carbon storage capacity [13,14].

Climate change is causing significant disruptions in many developing nations, particularly those whose economies heavily rely on climate-sensitive industries with limited adaptability [15]. The variability and trends in climate have profound effects on the environment and social development, which are crucial for supporting a growing human population [16]. Understanding these climatic trends is essential because numerous global challenges, including food insecurity, water scarcity, biodiversity loss, and health issues, are intrinsically linked to climate change [17]. Extensive research has been conducted to analyze climate trends across various regions and periods, to explore the causes of these trends, and to examine their effects on the environment and human societies [18].

Ethiopia, situated in the Sahel Region a zone known for its unpredictable climate fluctuations and irregular rainfall has been experiencing extreme temperatures, often leading to significant disasters [19]. Most of these disasters are climate-related, exacerbated by ecosystem degradation due to unregulated human activities. Poverty further intensifies the issue [20]. Other factors contributing to Ethiopia’s vulnerability to climate variability and change include its heavy dependence on rain-fed agriculture [21], underdeveloped water resources, rapid population growth, weak institutional frameworks, and a general lack of awareness [22]. Recent climate variability has posed substantial challenges to Ethiopia, affecting natural disasters, resource degradation, food security, water and energy supply, poverty alleviation, and sustainable development initiatives [23].

In recent decades, Ethiopia has experienced a temperature increase of approximately 0.37°C, indicating a shift in its climate [24]. Since the 1990s, there has been a notable decline in rainfall, significantly impacting the country’s water supply and agricultural productivity [25]. Both increased human activities and natural climate variability have played substantial roles in the observed changes in precipitation across Ethiopia [26]. Studies in Ethiopia [27–30] have highlighted the significant impact of climate change on crop productivity. According to [31], agricultural productivity in Ethiopia is projected to decline due to climate variability between 2030 and 2050, potentially increasing the nation’s dependence on food aid. This underscores the need for further research to identify observed climate changes and develop effective adaptation measures [32].

Previous studies on the Bilate watershed in Ethiopia have revealed significant impacts of LULC changes on hydrology, soil erosion, and crop production. Research by [33] indicates that agricultural expansion, deforestation, and population pressure have led to substantial deforestation and land degradation, thereby altering the region’s hydrology and increasing soil erosion. The conversion of forests and grasslands into agricultural lands has resulted in reduced soil fertility and productivity, exacerbating food insecurity [34]. Additionally, deforestation has decreased evapotranspiration, leading to higher temperatures and reduced rainfall, which exacerbates water scarcity and adversely affects agricultural productivity [35]. While these studies have extensively examined the impacts of LULC changes on hydrology, soil erosion, and agricultural productivity, there is a notable gap in research regarding the long-term impacts of LULC changes on climate change and variability. This research aims to address this gap by investigating the profound impacts of LULC changes on climate change and variability over time, thus filling the void left by previous research efforts. Therefore, this research work is intended to: (i) assess the spatiotemporal changes of LULC over the past 30 years (1994–2024) in the Bilate watershed, and (ii) investigate climate variability and trends over the Bilate watershed, thereby addressing the gaps left by previous research efforts.

This study is significant as it provides a comprehensive analysis of the long-term impacts of LULC changes on climate variability in the Bilate River Basin, a dimension that has been largely overlooked in previous research. By examining the interplay between LULC dynamics and climate trends over three decades, the study offers critical insights into how land management practices influence regional climate patterns. The findings will inform policymakers and stakeholders on the importance of sustainable land use strategies to mitigate adverse climate effects, safeguard water resources, and ensure agricultural sustainability in the face of ongoing environmental changes.

## 2. Method

### 2.1. Study area

The Bilate River Basin is located in Ethiopia, originating from the Gurage Mountains and draining into the Lake Abaya-Chamo watershed. It covers 5625 square kilometers and spans from the Ethiopian Highlands to the Rift Valley lowlands. The altitude ranges from 1,146 to 3,393 meters above sea level. Geographically, its location extends from 6° 36’N 38°00’E to 8°05’N 38°12’E (Fig 1).

**Fig 1:** Location map of the study area.

### 2.2. Data source

#### 2.2.1. Satellite data

To study and analyze LULC changes in the Bilate Watershed, multispectral satellite images of the area were acquired for four distinct years: 1994, 2004, 2014, and 2024. The temporal span of these images enables a comprehensive analysis of LULC dynamics over 30 years. Table 1 summarizes the acquisition details for each set of satellite images.

**Table 1:** Satellite data acquisition.

Year	Sensor type	Spatial Resolution	Acquisition Date	Source
1994	Landsat MSS	30m	12/1/1994	www.glovis.gov
2004	Landsat TM	30m	11/14/2004	www.glovis.gov
2014	Landsat 8 OLI/TIRS	30m	11/28/2014	www.glovis.gov
2024	Landsat 8 OLI/TIRS	30m	02/16/2024	www.glovis.gov

#### 2.2.2. Metrological data

For climate variability and trend analysis in the Bilate Watershed, meteorological data was obtained from the Ethiopian National Meteorological Agency (NMA). Data collection spanned five stations strategically distributed across the watershed’s three catchments. In the upper catchment, data was gathered from Fonko and Hossaina stations. Alaba Kulito and Durame stations were selected for the middle catchment, while Bodity station was used for the lower catchment. This distribution of meteorological stations ensures comprehensive coverage of the watershed, facilitating detailed analysis of climatic trends and variability across different altitudinal zones and land use areas.

#### 2.2.3. Reference data acquisition

The research conducted an accuracy assessment for the classified satellite images using a total of 300 Ground Control Points (GCPs). These GCPs were systematically collected from September 20, 2023, to October 28, 2024, ensuring comprehensive spatial coverage across five distinct LULC categories. The GCPs for the Settlement category were collected from impervious surfaces and roads in the towns of Durame, Hossaina, and Alaba Kulito. Forest GCPs were obtained through collaboration with the Bilate Watershed Authority. Bare land GCPs were sourced from open spaces predominantly covered with sand. Agricultural GCPs were gathered from various individual farmlands within the watershed. For the water body category, GCPs were referenced against lakes located in the Bilate catchment area.

### 2.3. Data preprocessing

Data preprocessing for both satellite and meteorological datasets involves several critical steps to ensure the data is accurate and suitable for analysis. For satellite data, the process includes radiometric and geometric corrections to adjust pixel values and align images with real-world coordinates, respectively. This is followed by an image sub-setting to focus on the Bilate Watershed, and cloud masking to exclude cloud-covered areas. For meteorological data, preprocessing begins with collecting data from five stations (Fonko, Hossaina, Alaba Kulito, Durame, and Bodity) and includes cleaning to handle missing values and outliers, homogenization for consistency, and temporal aggregation for trend analysis.

### 2.4. Data analysis

The overall methodology of the study is outlined in the flowchart (Fig 2). Following the preprocessing of satellite and meteorological data, the data analysis phase commenced. LULC classification was executed using the Google Earth Engine (GEE) platform, employing the Random Forest (RF) classification method to classify images for the years 1994, 2004, 2014, and 2024 within the river basin. Post-classification, an accuracy assessment was carried out to evaluate how well the classification results matched the ground reality, utilizing the collected GCP. Subsequently, change detection analysis was performed to identify land use transitions and to determine the dynamics over the 30 years. This analysis helped in understanding which land use categories were converted into others and the extent of these changes. In parallel, climate variability and trend analysis were conducted using the meteorological data for the river basin. The Mann-Kendall test was applied to assess trends in the climatic data. For analyzing climate variability, statistical measures such as the coefficient of variation were employed. Additionally, for drought vulnerability analysis, the Standardized Precipitation Index (SPI) and Standardized Temperature Index (STI) were utilized. These indices helped in identifying periods of drought and assessing their severity.

**Fig 2:** Methodological flowchart.

#### 2.4.1. Land use land cover classification

The Random Forest (RF) classification method was used for image classification. The choice of employing the Random Forest (RF) machine learning approach for land cover classification is driven by its recognized superiority in achieving high classification accuracy. Particularly within Google Earth Engine (GEE), RF is widely adopted for both classification and regression tasks, as emphasized by the work of [36]. This algorithm is selected for its capacity to provide robust and accurate predictions through an ensemble learning paradigm. The RF process involves the generation of multiple decision trees, each constructed based on random subsets of features, thereby enhancing diversity and robustness. Bootstrapping initiates the classification procedure by creating varied sets of decision trees through random subsampling of the dataset with replacement. During tree construction, feature randomization is introduced to consider only subsets of features at each node, mitigating the risk of overfitting and enhancing model stability. In classification tasks, the ultimate prediction is determined through a majority voting mechanism among the individual trees, constituting an ensemble decision-making process expressed mathematically in Eq 1. The percentage of training and test data in the RF model is typically allocated around 70–80% for training and 20–30% for testing, ensuring a balance between model training and evaluation [37]. Hyperparameters, such as the number of trees, maximum tree depth, and features considered at each split, play a crucial role in RF model performance. The optimum values for these parameters are determined through hyperparameter tuning, with techniques like random search exploring the parameter space. The specific values depend on the characteristics of the dataset and the complexity of the land cover classification task.


D={(x1,y1),(x2,y2),….,(xn,yn)} (1)

Where D is the bootstrapped dataset, xi stands as a vector of M feature values for the ith sample, and yi is the corresponding class label for classification.

#### 2.4.2. Accuracy assessment

The accuracy assessment of classified land cover maps is a crucial step in ensuring the reliability of satellite-based classifications. For the accuracy assessment, GPS data, existing land cover maps, and Google Earth imagery were employed. Once validation points from various sources are acquired, accuracy assessment statistics, including User Accuracy, Producer Accuracy, and Overall Accuracy, were computed (Eqs 2–4). These statistics provide quantitative measures of the classification’s performance, offering insights into the reliability and precision of the classified land cover maps over the specified time frame. This comprehensive validation strategy helps overcome challenges related to ground data accessibility and ensures the robustness of the land cover classification results.


$$OA=\frac{Number\;of\;correctly\;classified\;pixel}{Total\;number\;of\;pixels}*100$$ (2)

$$UA_{i}=\frac{Number\;of\;correctly\;classified\;pixel\;for\;class\;i}{Total\;number\;of\;pixels\;classified\;as\;class\;i}*100$$ (3)

$$PA_{i}=\frac{Number\;of\;correctly\;classified\;pixel\;for\;class\;i}{Total\;number\;of\;pixels\;of\;class\;i}*100$$ (4)

#### 2.4.3. Climate variability and trends

To investigate the evolution of climatic characteristics over time, various analytical approaches are employed. The Standardized Precipitation Index (SPI) assesses changes in precipitation patterns by examining the frequency and intensity of precipitation events, providing insights into trends and variability. The Mann-Kendall (MK) trend test is utilized to detect significant climate trends in time series data, identifying monotonic increases or decreases that indicate long-term changes. Concurrently, the Standardized Temperature Index (STI) measures temperature variability across a study area’s observed time scale, offering a standardized metric for comparing temperature fluctuations.

*2*.*4*.*3*.*1 Standardize Precipitation Index (SPI)*. The Standard Precipitation Index (SPI) is a widely utilized tool for assessing and monitoring precipitation anomalies over different time scales, crucial for identifying periods of drought or excess rainfall. The SPI standardizes precipitation data, allowing for meaningful comparisons across diverse climates and geographical locations. This index can be determined using the following equation (Eq 5):

$$Z=\frac{Xi-\bar{Xi}}{S}$$ (5)

Z is the Standardized Precipitation Index (SPI), representing the deviation of annual precipitation Xi from the mean (Xi) of the historical record, scaled by the standard deviation S of the annual precipitation.

*2*.*4*.*3*.*2 Standardize Temperature Index (STI)*. The Standardized Temperature Index (STI) is a statistical measure used to assess and quantify temperature anomalies over a specific period. It is particularly useful in identifying and evaluating periods of unusually high or low temperatures, thereby aiding in the analysis of climate variability and trends (Eq 6). The STI is analogous to the Standardized Precipitation Index (SPI), which is used for drought assessment based on precipitation data.


$$STI=\frac{Ti-\mu }{\sigma }$$ (6)

Where; Ti is the temperature for a specific period (seasonal), μ is the mean temperature over a reference period, σ is the standard deviation of the temperature over the same reference period.

*2*.*4*.*3*.*3 Mann Kendall Test*. The Mann-Kendall Trend Test assesses monotonic trends in time-series data, such as temperature and precipitation from 1994 to 2024, using metrological records. It calculates the Mann-Kendall test statistic S, which evaluates the sum of signs of pairwise differences in the data series. The variance Var (S) considers tied groups within the data, adjusting for any non-independence. The resulting standard normal test statistic Z is derived from S and Va (S), indicating the significance of observed trends: positive Z values denote increasing trends, negative values indicate decreasing trends, and values exceeding critical thresholds suggest statistical significance (Eqs 7–9). This non-parametric approach accommodates data of all distributions and is crucial for detecting climate and environmental changes over time reliably [38]:

$$Z=\left[\begin{array}{l} \frac{S-1}{\sqrt{V(S)}},\;for\;S>0\\ 0\;for\;s=0\\ \frac{S+1}{\sqrt{V(S)}},\;for\;S<0 \end{array}\right]$$ (7)

$$S=\sum_{i=1}^{n-1}\sum_{j=i+1}^{n}sign(X_{j}-X_{i})$$ (8)

$$sign=\left[\begin{array}{c} 1\;for\;(X_{j}-X_{i})>0\\ 0\;for\;(X_{j}-X_{i})=0\\ -1\;for\;(X_{j}-X_{i})<0 \end{array}\right]$$ (9)

$$V(S)=\frac{1}{18}\left[n(n-1)(2n+5)-\sum_{p=1}^{q}t_{p}(t_{p}-1)(2t_{p}+5)\right]$$ (10)

## 3. Result

### 3.1. Spatiotemporal dynamics of LULC over the past 30 years (1994–2024)

Between 1994 and 2004, the Bilate River Basin saw a significant reduction in forest cover (Fig 3), dropping from 284,048.74 hectares (50.50% of the basin) to 215,361.21 hectares (38.29%). This represents a substantial loss of 68,687.53 hectares, highlighting extensive deforestation. Conversely, agricultural land expanded considerably, from 265,283.26 hectares (47.16%) to 331,394.54 hectares (58.91%), indicating a growth of 66,111.28 hectares. The built-up areas also increased markedly, from a mere 4.14 hectares to 3,013.64 hectares (0.54%), driven by urbanization and infrastructure development. The area of water bodies saw a modest increase from 769.95 hectares (0.14%) to 1,040.32 hectares (0.18%), while bare land decreased slightly from 12,375.51 hectares (2.20%) to 11,706.47 hectares (2.08%) (Table 2). From 2014 to 2024 (Fig 4), the trends observed earlier continued, with forest cover further reducing from 210,786.52 hectares (37.47%) to 163,974.43 hectares (29.15%), a loss of 46,812.09 hectares. Agricultural land, which had seen a slight decline by 2014, increased again from 329,668.21 hectares (58.61%) to 341,078.85 hectares (60.64%), marking an addition of 11,410.64 hectares. Bare land saw a dramatic increase from 15,134.67 hectares (2.69%) to 48,799.57 hectares (8.68%), highlighting severe land degradation issues. The built-up area continued to grow significantly from 3,504.45 hectares (0.62%) to 7,251.68 hectares (1.29%), reflecting ongoing urbanization. Water bodies, however, experienced a reduction from 3,382.87 hectares (0.60%) to 1,331.32 hectares (0.24%), indicating possible issues with water management or conservation.

**Fig 3:** Land cover maps of Bilate Watershed between 1994–2004.

**Fig 4:** Land cover maps of Bilate Watershed between 2014–2024.

**Table 2:** Land use land cover dynamics over the past 30 years (1994–2024).

	1994		2004		2014		2024	
Class Name	Area	%	Area	%	Area	%	Area	%
Forest	284048.74	50.50	215361.21	38.29	210786.52	37.47	163974.43	29.15
Water Body	769.95	0.14	1040.32	0.18	3382.87	0.60	1331.32	0.24
Bare land	12375.51	2.20	11706.47	2.08	15134.67	2.69	48799.57	8.68
Built up	4.14	0.00	3013.64	0.54	3504.45	0.62	7251.68	1.29
Agriculture	265283.26	47.16	331394.54	58.91	329668.21	58.61	341078.85	60.64
Total	562481.60	100.00	562516.18	100.00	562476.72	100.00	562435.85	100.00

### 3.2. Rate of change

From 1994 to 2004, the Bilate River Basin underwent notable changes in land use and land cover, reflecting significant environmental and socio-economic shifts. Forest areas experienced a substantial decline, with an average annual loss of 686.9 hectares, largely driven by logging, agricultural expansion, and urbanization [33]. This period also saw a modest increase in water bodies by 27.01 hectares per year, likely due to improved watershed management and natural hydrological processes (Table 3). Concurrently, bare land decreased by 66.95 hectares annually, suggesting successful soil conservation and land reclamation efforts. The built-up area expanded rapidly at a rate of 300.47 hectares per year, indicating robust population growth and infrastructural development. Agricultural land grew dramatically by 6,611 hectares annually, underscoring the escalating demand for food production and land conversion [39,40]. These changes highlight the complex interplay between natural processes and human activities, necessitating sustainable land management practices to mitigate adverse environmental impacts.

**Table 3:** Rate change of land use land cover changes from 1994–2024.

	1994–2004	2004–2014	2014–2024	1994–2024
Forest	-686.9	-457.5	-4,681.20	-4,002.49
Waterbody	27.01	130.2	-20.51	18.7
Bare land	-66.95	342.8	336.65	40.47
Built up	300.47	49.1	24.3	241.42
Agricultures	6,611	-172.6	1141	2526.2

The decade from 2004 to 2014 marked further dynamic shifts in the Bilate River Basin’s land cover. The rate of forest loss, although still significant, slowed to 457.5 hectares per year, possibly due to initial conservation efforts and changes in land use policies [41]. Water bodies saw a more pronounced increase, growing by 130.2 hectares annually, which can be attributed to enhanced water management and conservation measures. However, bare land began to increase significantly at a rate of 342.8 hectares per year, indicating rising deforestation and land degradation issues. The expansion of built-up areas slowed to 49.1 hectares per year, reflecting more stringent urban planning and land use regulations. Interestingly, agricultural land decreased 172.6 hectares annually, potentially due to soil degradation, reduced fertility, and conversion of agricultural land to other uses. These trends underscore the necessity for ongoing and improved land management strategies to balance development with environmental sustainability.

Between 2014 and 2024, the trends in land use and land cover change became even more pronounced, with significant implications for the region’s environmental and socio-economic landscape. Forest areas continued to decline sharply, with an alarming annual loss rate of 4,681.2 hectares, exacerbating issues such as habitat loss, biodiversity decline, and increased carbon emissions. The area covered by water bodies decreased slightly by 20.51 hectares per year, raising concerns about water resource management and climate change impacts [42]. Bare land expanded at a rate of 336.65 hectares annually, reflecting ongoing land degradation and deforestation pressures. Meanwhile, the growth rate of built-up areas slowed further to 24.3 hectares annually, suggesting more controlled and sustainable urban development. Agricultural land began to increase again at a rate of 1,141 hectares per year, indicating efforts in land recovery and sustainable farming practices. These changes highlight the urgent need for comprehensive land management strategies, environmental conservation initiatives, and sustainable development practices to address the complex challenges facing the Bilate River Basin [43].

### 3.3. Accuracy assessment

The accuracy assessment results for land cover classification in the Bilate River Basin from 1994 to 2024 indicate varying levels of producer and user accuracy across different land cover types, with overall accuracy and kappa values reflecting improvements over time. In 1994, the overall accuracy was 0.63 with a kappa value of 0.52, indicating moderate agreement. By 2004, overall accuracy increased to 0.67 and the kappa value to 0.59, showing improved classification reliability. The trend continued in 2014, with overall accuracy reaching 0.74 and a kappa of 0.68, reflecting substantial agreement. In 2024, the overall accuracy slightly declined to 0.71, with a kappa value of 0.65, still indicating substantial agreement. Notably, the accuracy of forest classification fluctuated, with the highest user accuracy of 1.00 observed in both 1994 and 2024, while water bodies and built-up areas showed significant variability in accuracy over the years (Table 4).

**Table 4:** Accuracy assessment results (1994, 2004, 2014 and 2024).

	1994		2004		2014		2024	
Land cover	Producer	User	Producer	User	Producer	User	Producer	User
Forest	0.67	1.00	0.68	0.40	0.64	0.50	0.68	1.00
Water Body	0.76	0.86	0.68	0.95	0.96	0.79	1.00	0.85
Bare land	0.60	0.50	1.00	0.83	0.92	0.72	0.96	0.44
Built up	0.36	0.26	0.95	0.49	0.65	0.62	0.75	0.60
Agricultures	0.80	0.92	0.80	1.00	0.70	1.00	0.90	1.00
Overall	0.63		0.67		0.74		0.71	
Kappa	0.52		0.59		0.68		0.65	

### 3.4. Climate variability and trends

The seasonal rainfall variations across the Bilate watershed from 1994 to 2024 demonstrate distinct trends in each catchment. In the upper catchment, winter, autumn, and summer exhibit significant negative trends in rainfall (Kendall’s tau: -0.315, -0.300, and -0.305, respectively, all with p-values < 0.01), indicating a decline in precipitation, while spring shows no significant trend. In the middle catchment, spring displays a significant positive trend (tau: 0.459, p < 0.0001) with an increase in rainfall, whereas summer has a marginally non-significant negative trend (tau: -0.193, p = 0.078), and winter and autumn show no significant trends. The lower catchment sees significant positive trends in spring (tau: 0.535, p < 0.0001) and autumn (tau: 0.244, p = 0.025), indicating increased rainfall, while winter and summer show no significant changes (Table 5).

**Table 5:** Seasonal rainfall variation across each catchment in the Bilate watershed.

	Season	Kendall’s tau	p-value	Sen’s slope
Upper Catchment	Winter	-0.315	0.004*	-3.819
	Autumn	-0.300	0.006*	-7.972
	Summer	-0.305	0.005*	-7.117
	Spring	-0.086	0.438	-0.934
Middle Catchment	Winter	-0.084	0.445	-0.740
	Autumn	0.054	0.629	1.540
	Summer	-0.193	0.078	-3.515
	Spring	0.459	**< 0.0001**	6.058
Lower Catchment	Winter	0.143	0.192	1.630
	Autumn	0.244	**0.025**	6.424
	Summer	0.022	0.849	0.615
	Spring	0.535	**< 0.0001**	7.689

Fig 5 shows the seasonal trends of rainfall over three catchments from 1994 to 2024. In all three catchments (Upper, Middle, and Lower), autumn consistently exhibits the highest rainfall, followed by summer, with winter and spring having considerably lower rainfall. Notably, there is significant interannual variability in rainfall, especially in autumn and summer, with peaks around the early 2000s and mid-2010s. The Upper catchment (a) and Middle catchment (b) have relatively similar rainfall patterns, while the Lower catchment (c) shows more pronounced peaks in autumn rainfall, particularly around 2015.

**Fig 5:** Seasonal trends of rainfall over the three catchments (a) Upper catchment, (b) Middle catchment, (c) Lower catchment.

Table 6 presents the seasonal temperature variation across the Upper, Middle, and Lower catchments in the Bilate watershed, showing Kendall’s tau, p-value, and Sen’s slope for each season. In the Upper catchment, all seasons exhibit significant positive trends in temperature, with autumn showing the highest Kendall’s tau (0.429) and the smallest p-value (<0.0001), indicating a strong and significant upward trend. Winter, summer, and spring also show significant positive trends with p-values below 0.01. In contrast, the Middle catchment shows a significant positive trend only in summer (tau = 0.254, p = 0.020), while other seasons do not exhibit significant trends. The Lower catchment shows no significant trends in any season, with all p-values above 0.1, and some seasons even showing negative Kendall’s tau values, indicating no consistent temperature increase. Overall, the Table 6 indicate a clear and significant warming trend in the Upper catchment across all seasons, a moderate trend in the Middle catchment during summer, and no significant trends in the Lower catchment.

**Table 6:** Seasonal temperature variation across each catchment in Bilate watershed.

	Season	Kendall’s tau	p-value	Sen’s slope
Upper Catchment	Winter	0.341	0.002*	0.029
	Autumn	0.429	< 0.0001*	0.030
	Summer	0.414	0.000*	0.018
	Spring	0.302	0.006*	0.022
Middle Catchment	Winter	-0.011	0.928	-0.001
	Autumn	0.116	0.291	0.013
	Summer	0.254	**0.020**	0.016
	Spring	0.034	0.762	0.003
Lower Catchment	Winter	-0.166	0.129	-0.014
	Autumn	0.078	0.479	0.006
	Summer	0.165	0.132	0.010
	Spring	-0.113	0.301	-0.008

Fig 6 illustrates the seasonal temperature trends across the three catchments (a) Upper, (b) Middle, and (c) Lower catchments from 1994 to 2024. In the Upper catchment (a), there is a noticeable upward trend in temperatures across all seasons, with winter showing the highest temperatures, followed by autumn, summer, and spring. This is justified by Table 6, where significant positive trends were found in all seasons for the Upper catchment, with p-values below 0.01, indicating a consistent increase in temperature. The Middle catchment (b) also exhibits a general upward trend, particularly in winter, although the seasonal variations are less pronounced than in the Upper catchment. This aligns with Table 6, which shows a significant positive trend only in summer, indicating less overall temperature increase. The Lower catchment (c) demonstrates higher overall temperatures compared to the other catchments, with winter temperatures peaking higher than other seasons. However, the trends in the Lower catchment are less consistent, with more variability, especially in autumn and spring, as evidenced by Table 6, where no significant trends were found in any season. Thus, the graphs indicate a general warming trend across all catchments, with winter consistently being the warmest season.

**Fig 6:** Seasonal trends of temperature over the three catchments (a) Upper catchment, (b) Middle catchment, (c) Lower catchment.

The observed differences in temperature trends across the three catchments can be explained by several key factors. Variations in land use, such as deforestation and agriculture, can impact local temperatures. Reduced vegetation in the middle and upper catchments can lead to higher surface temperatures, while the lower catchment might retain more moisture and have cooler temperatures due to better vegetation cover. This relationship between land use and temperature is well documented in studies like those by [44,45]. Anthropogenic climate change affects temperature patterns differently across elevations. Lower catchments may experience more significant warming due to urbanization and increased greenhouse gas emissions, while upper catchments might show mixed trends due to the varying impacts of global warming on high-altitude climates. The [46–49] reports provide comprehensive evidence on how global warming is altering temperature patterns worldwide.

### 3.5. Drought Severity Index (DSI)

#### 3.5.1. Standardized Precipitation Index (SPI)

The updated Fig 7 depicts the SPI for the upper, middle, and lower catchments from 1994 to 2024, illustrating the variability in drought conditions. The upper catchment exhibits significant fluctuations, with notable wet periods around 1995, 2010, and 2020, where SPI values exceed 2.0, and severe droughts around 2000 and 2015, where values drop below -1.0. This variability suggests a high sensitivity to climatic changes, likely influenced by its altitude and orographic effects. The middle catchment shows similar trends but with moderated extremes, indicating less sensitivity compared to the upper catchment. Noteworthy wet periods are observed around 1995 and 2010, with significant droughts around 2000 and 2015. The lower catchment displays the least variability, with less extreme SPI values throughout the observed period. Significant wet conditions are seen around 1995 and 2020, while droughts are less severe than in the other catchments. These patterns reflect the lower catchment’s more stable climatic influences and lower altitude. The overall trends across all catchments highlight an increasing frequency of extreme precipitation events in recent years, potentially due to anthropogenic climate change [47]. Additionally, land use changes such as deforestation and urbanization in the middle and lower catchments may contribute to the moderated SPI values observed [50].

**Fig 7:** Standardized Precipitation Index (SPI) over the three catchments.

#### 3.5.2. Standardized Temperature Index (STI)

The STI shows significant temperature anomalies and their variations across the upper, middle, and lower catchments from 1994 to 2024, revealing unique climatic dynamics in each region. The upper catchment shows pronounced variability from 1994 to 1999 with alternating warm and cool phases, attributed to its higher elevation, followed by more stable conditions from 1999 to 2004, except for a warm period around 2003–2004. Post-2004, increased temperature variability indicates rising anomalies likely due to broader climatic changes. The middle catchment experiences similar but less extreme variations during the same initial period, with stability between 1999 and 2004, and moderate variability thereafter, aligning with trends in the upper catchment. The lower catchment, influenced by its lower altitude, exhibits moderate variability from 1994 to 1999 and a significant warm anomaly around 2003–2004, with increasing variability from 2004 onwards, reflecting broader climatic influences observed in the upper and middle catchments (Fig 8).

**Fig 8:** Standardized Temperature Index (STI) over the three catchments.

### 3.6. Interplay between land use land cover change and climate variability

The association between land cover change and climate variability in the Bilate River Basin over the past 30 years demonstrates a complex interplay where anthropogenic activities and natural climatic shifts exacerbate environmental changes. The significant reduction in forest cover, which dropped from 284,048.74 hectares in 1994 to 163,974.43 hectares in 2024, is linked to increased deforestation driven by agricultural expansion and urbanization. This loss of forest area correlates with rising temperatures and altered precipitation patterns. Studies have shown that deforestation leads to reduced evapotranspiration and changes in surface albedo, contributing to local and regional climate warming [51,52]. The concurrent increase in agricultural land from 265,283.26 hectares to 341,078.85 hectares has further disrupted the local climate by increasing land surface temperatures due to the replacement of forests with cropland [53].

Climate variability, characterized by significant seasonal changes in rainfall and temperature across different catchments, further influences land cover dynamics. The observed decrease in seasonal rainfall in the upper catchment, coupled with an increase in temperature, suggests a feedback loop where reduced forest cover exacerbates drought conditions, which in turn inhibits forest regrowth and promotes land degradation. The rise in bare land from 12,375.51 hectares in 1994 to 48,799.57 hectares in 2024 underscores this degradation. The variability in rainfall patterns, with significant positive trends in the lower catchment’s spring and autumn rainfall, contrasts with the significant negative trends in the upper catchment’s winter and autumn rainfall, reflecting how land cover changes can differentially impact microclimates within a watershed [48,54].

The shifts in land cover also impact drought severity indices such as the SPI and STI. The upper catchment, experiencing pronounced variability in these indices, highlights its sensitivity to both climatic changes and land cover modifications. Deforestation and agricultural expansion have likely increased the region’s vulnerability to extreme climatic events, evidenced by the increased frequency of both severe droughts and wet periods in recent years. This pattern aligns with global studies indicating that land use changes, such as deforestation, can significantly amplify climate extremes by altering hydrological cycles and surface energy balances [47,50,55]. Hence, the observed trends in the Bilate River Basin underscore the critical need for integrated land and climate management strategies to mitigate adverse environmental impacts.

## 4. Discussion

The significant decline in forest cover in the Bilate watershed from 50.4% in 1994 to 29.1% in 2024 is indicative of widespread deforestation and forest degradation, aligning with trends observed across Ethiopia and other parts of Africa. Studies such as those by [56] attribute this forest loss to agricultural expansion and population pressure. Similarly, [57] noted that deforestation in Ethiopia is often driven by the need for agricultural land and fuelwood, with long-term implications for biodiversity and climate change. The increase in agricultural land from 47.1% to 60.6% over the study period in the Bilate watershed reflects a common trend in many developing regions, driven by the need to meet the food demands of a growing population. This expansion, as reported by [58,59], poses a significant threat to sustainable land management by converting forested and marginal lands into agricultural use.

The growth of built-up areas in the Bilate watershed from 0.007% to 1.3% reflects significant urban development driven by economic growth and population increase, a trend mirrored in many rapidly developing regions [9,42]. Urbanization often leads to the conversion of agricultural and natural lands into urban infrastructure, with profound implications for local ecosystems and biodiversity. The variability in the extent of water bodies in the Bilate watershed, with an overall reduction in recent years, highlights the impact of environmental changes and water management practices, as observed in other watersheds studied by [60,61]. Additionally, the increase in bare land from 2.2% to 8.6% suggests issues such as soil erosion and land degradation, consistent with findings from studies by [41,42]. These trends underscore the importance of implementing sustainable land management practices and soil conservation measures to combat soil erosion and maintain land productivity, as emphasized by [62].

The findings of this research indicate that the middle and lower catchments, more affected by human activities such as deforestation and urbanization, show moderated SPI values. This is consistent with [63,64], which confirms that land use changes can significantly alter local climates by affecting surface albedo, evaporation rates, and atmospheric circulation. Studies by [65,66] further emphasize the impact of agricultural expansion and urban development in Ethiopia, which aligns with the observed trends in the Bilate watershed’s middle and lower catchments. Studies by [48,49] report increased climate variability, with more frequent and severe weather events like droughts and heavy rainfall. The research findings of more frequent extreme weather events in the Bilate watershed corroborate this, showing increased SPI variability. Additionally, research by [61,67–69] highlight similar trends of declining rainfall during critical periods in other parts of Ethiopia, reinforcing global patterns. The research findings mention significant seasonal rainfall variations, with the lower catchment showing increases during spring and autumn, and the upper catchment experiencing decreases during monsoon months. This aligns with studies, such as those by and [70], which emphasizes the impact of changing seasonal weather patterns on regional hydrology. Other studies like those by [28,71] confirm these trends, noting similar seasonal variations in rainfall across different Ethiopian regions.

## 5. Conclusion

The study of the Bilate River Basin over the past three decades reveals significant changes in LULC with profound implications for the region’s climate and environment. Forest cover has dramatically decreased from 1994–2024, showing extensive deforestation, while agricultural land has expanded over the past 30 years, driven by the need for more cultivable land to support the growing population. Urbanization is evident in the substantial growth of built-up areas, which contributes to local climate changes, such as the heat island effect and increased greenhouse gas emissions. Climatic trends analyzed using the Mann Kendall test reveal increasing frequency and intensity of extreme weather events, underscoring the basin’s sensitivity to climatic changes driven by natural variability and human activities. Temperature trends show significant anomalies, particularly in the upper catchment due to its anthropogenic activities, with moderated but notable variations in the middle and lower catchments. These findings highlight the urgent need for sustainable land management practices, effective water management, and conservation strategies to address deforestation, urbanization, and agricultural expansion. Integrated approaches to land and climate management are essential to foster sustainable development and enhance the resilience of the Bilate River Basin to future climatic shifts.
